The article "The mouse complement regulator CD59b is significantly expressed only in testis and plays roles in sperm acrosome activation and motility" was retracted in 2014. Reason: manipulated images.

# The mouse complement regulator CD59b is significantly expressed only in testis and plays roles in sperm acrosome activation and motility

**DOI:** 10.1016/j.molimm.2007.05.011

**Published:** 2008-01

**Authors:** Rossen M. Donev, Baalasubramanian Sivasankar, Masashi Mizuno, B. Paul Morgan

**Affiliations:** Department of Medical Biochemistry and Immunology, School of Medicine, Cardiff University, Cardiff CF14 4XN, UK

**Keywords:** Mouse, CD59a, CD59b, Complement, Reproductive immunology, Acrosome

## Abstract

In mouse, genes encoding complement regulators CD55 and CD59 have been duplicated. The first described form of CD59, CD59a, is broadly distributed in mouse tissues, while the later identified CD59b was originally described as testis specific. Subsequent studies have been contradictory, some reporting widespread and abundant expression of CD59b. Resolution of the distribution patterns of the CD59 isoforms is important for interpretation of disease studies utilising CD59 knockout mice. Here we have performed a comprehensive distribution study of the CD59 isoforms at the mRNA and protein levels. These data confirm that expression of CD59b is essentially restricted to adult testis; trace expression in other tissues is a consequence of contamination with blood cells, shown previously to express CD59b at low level. In testis, onset of expression of CD59b coincided with puberty and was predominant on the spermatozoal acrosome. Ligation of CD59b, but not CD59a, markedly reduced spermatozoal motility, suggesting a specific role in reproductive function.

## 1 Introduction

CD59, a broadly distributed glycosyl phosphatidylinositol (GPI)-anchored protein, is the principal regulator of complement membrane attack complex (MAC) assembly on cell membranes (Meri et al., 1990). A decade ago, we identified the mouse analogue of CD59 and showed that it was broadly distributed on cells and tissues (Powell et al., 1997). Deletion of the gene encoding mouse CD59 caused minimal disturbance in unchallenged animals but markedly enhanced susceptibility to complement-driven pathologies (Holt et al., 2001; Turnberg et al., 2003, 2004; Lin et al., 2004; Mead et al., 2004; Williams et al., 2004). Others demonstrated that the gene encoding CD59 is duplicated in the mouse; the protein products of these two genes were then termed CD59a for the first described, and CD59b for the product of the new gene (Qian et al., 2000). In this first report, it was stated that CD59b message was significantly expressed only in testis. We developed monoclonal antibodies specific for CD59a and CD59b, enabling us to confirm the broad distribution of CD59a and testis restricted expression of CD59b at the protein level; we concluded that CD59a was the principle regulator of MAC assembly in mouse tissues (Harris et al., 2003). This conclusion was challenged in a re-analysis of the pattern of distribution of mRNA encoding the two forms of CD59; these studies suggested that both CD59a and CD59b were broadly expressed in the mouse and contended that the latter was the major regulator of MAC in the mouse (Qin et al., 2003). These contentions were bolstered by the demonstration that deleting the gene encoding CD59b in mice caused a severe, spontaneous phenotype with anaemia, platelet dysfunction and fertility problems. In light of these data we reassessed the distribution patterns at protein and mRNA levels using a combination of specific monoclonal antibodies and shared primers for PCR in high sensitivity assays (Baalasubramanian et al., 2004). These analyses confirmed our earlier work showing that CD59a was broadly expressed while significant expression of CD59b was restricted to testis. Trace amounts of CD59b message and protein were detected in erythrocytes but quantitative assays of protein expression showed that CD59b expression on erythrocytes was less that 5% that of CD59a. Further, we confirmed that CD59a was dominant in protection of erythrocytes from MAC lysis. The findings of these painstaking studies have recently been challenged yet again (Qin et al., 2006). The appropriateness of the techniques used and specificity of probes and primers have all been questioned. These authors concluded that CD59b was broadly expressed and an important regulator of MAC assembly on erythrocytes and in tissues.

We, and others, are using CD59a knockout mice in disease models to explore roles of MAC based on our evidence that CD59a is the principal regulator of the MAC in most tissues. If CD59b is indeed widely distributed then the value of studies in CD59a knockouts is in question. It is therefore essential that we test the evidence. Here using multiple methods we revisit these published studies and undertake new analyses to explore the expression patterns of CD59a and CD59b at the mRNA and protein level. We conclude that expression of CD59b at the mRNA and protein level is essentially absent in all tissues other than testis. Low level expression on blood cells was confirmed and trace detection of mRNA in tissues was shown to be likely due to blood contamination. We further analysed expression of CD59b in testis and showed that expression coincided with onset of puberty and was restricted to spermatozoa and their immediate precursors. Ligation of CD59b on spermatozoa with monoclonal antibody markedly inhibited sperm motility, suggesting a specific role in reproductive function.

## 2 Materials and methods

### 2.1 Mice

Adult (8–16 weeks) and infant (1–5 weeks; pre-puberty) male mice, and embryos (day 5, 10 and 15) from C57BL/6(H-2^b^) background mice were used in our investigation. All experimental procedures were performed in compliance with Home Office and local ethics committee regulations. *cd59a*−/− mice generated as described previously (Holt et al., 2001), and back-crossed 10 generation onto the same background were used as controls.

### 2.2 Antibodies and reagents

Rat anti-mouse CD59a (CD59a.1; IgG1) was generated in house (Harris et al., 2003). Mouse anti-mouse CD59b (CD59b.2; IgG1) was also made and characterized in house (Baalasubramanian et al., 2004). Separate aliquots of CD59a.1 and CD59b.2 were labelled with NHS-biotin (Sigma–Aldrich, Gillingham, Dorset, UK) and FITC-NHS (Perbio Science UK Ltd., Cramlington, UK) according to manufacturer's protocols. As negative controls, rat IgG1 and mouse IgG1 (purified in-house) were labelled in the same manner. FITC-labelled streptavidin was purchased from DAKO (Ely, Cambridgeshire, UK). HRPO-labeled donkey anti-rat IgG and HRPO-labeled donkey anti-mouse IgG were purchased from Jackson ImmunoResearch Europe (Newmarket, Suffolk, UK).

### 2.3 Semi-quantitative RT-PCR

Total RNA was purified from all investigated mouse tissues using GenElute kit (Sigma–Aldrich) and controlled for DNA contamination by RT-PCR without using reverse transcriptase and employing a β-actin specific primer pair (Table 1). Only samples that did not show amplification were used in all analyses. Aliquots of these RNAs (1 μg each) were reverse transcribed using random hexamers and multiscribe reverse transcriptase according to the manufacturer's instructions (Applied Biosystems, Warrington, UK). Primer pairs specific for either CD59a or CD59b were as described by Qin et al. (2006), and a new primer pair common for both CD59a and b and amplifying a sequence in exon 4 comprising 199 bp for CD59a and 162 bp for CD59b, were used in the subsequent amplifying reactions for detection of CD59a and CD59b mRNAs (Table 1). Either 25 or 35 amplification cycles were used, except where attempting simultaneous detection of both mRNAs when 40 cycles were performed. Amplified products were separated either in 1% agarose or in 5% poly-acrylamide gels (PAAG). To obtain semi-quantitative data for expression of the two genes, we used as templates either 2 μl of the original cDNA, or a series of dilutions as indicated in figures. Gels were scanned and band intensity was measured by densitometry using Quantity One 4.3.0 software (BioRad, Hemel Hempstead, Hertfordshire, UK). The quantifications were carried out in triplicate and means and errors calculated.

### 2.4 Quantitative real-time PCR analysis

The cDNAs from testis and liver prepared as described for the semi-quantitative RT-PCR, were subject to a Taqman assay as described previously (Baalasubramanian et al., 2004). One of the primer pairs was as described previously (Baalasubramanian et al., 2004), a perfect match for the sequence of CD59a mRNA and with a single internal nucleotide mismatch to CD59b mRNA; the second set was a perfect match for the same sequence in CD59b and with a single internal nucleotide mismatch to CD59a (Table 1).

To measure the relative number of mRNA copies for CD59b in liver, perfused liver and testis we used the primer pair reported by Qin et al. (2006) to specifically amplify CD59b in a quantitative PCR (QPCR). Because these primers were not designed specifically for this assay, they did not meet the optimal annealing temperature requirements. To correct for this anomaly, the standard amplification programme was modified to include a pre-annealing step at 56 °C for 20 s prior to the extension phase.

Primers were designed to β-actin (Table 1) as an internal control for normalization of starting cDNA levels. Quantitative PCR was performed on ABI PRISM 7000 using either TaqMan Universal PCR Master Mix or SYBR Green PCR Master Mix according to the manufacturer's instructions (Applied Biosystems) with 50 cycles of amplification.

### 2.5 Preparation of tissue lysates

To obtain tissue lysates, freshly harvested mouse organs were immediately chilled and homogenized with ice-cold lysis buffer (PBS containing 2% NP40, 1 mM phenylmethylsulfonyl fluoride, 10 mM EDTA, 1 μg/ml leupeptin, and 1 μg/ml pepstatin; 1 g of tissue/1.5 ml of buffer) and incubated for 60 min on ice. Insoluble debris was removed by centrifugation (5000 × *g*, 15 min at 4 °C) and the supernatants stored in aliquots at −80 °C until use. In some experiments the mouse was perfused with saline at the time of sacrifice to reduce blood contamination in harvested organs.

### 2.6 SDS-PAGE and Western blot analysis

Lysates were mixed 1:1 with sample buffer for SDS-PAGE and separated under non-reducing conditions in 15% gels. Separated proteins were transferred onto nitrocellulose membranes (Schleicher & Schuell, London, UK), and membranes blocked with 5% (w/v) non-fat milk in PBS (PBS-M). Membranes were then probed with the primary mAb diluted in PBS-M, washed in PBS containing 0.1% Tween-20 (PBS-T), then probed with HRPO-conjugated donkey anti-rat Ig in PBS-M to detect the rat anti-CD59a or HRPO-conjugated donkey anti-mouse Ig (Jackson) to detect the mouse anti-CD59b. After further washing in PBS-T, bands were developed using ECL (Perbio Science UK Ltd.) and captured on autoradiographic film (Kodak Ltd., Hemel Hempstead, Hertfordshire, UK).

### 2.7 Spermatozoa preparation and analysis

Motile cauda epididymal spermatozoa were obtained by a ‘swim-up’ technique as previously described (Mizuno et al., 2004, 2005). Briefly, two cauda epididymi from an adult C57BL/6 mouse were roughly minced in 1 ml of DMEM (Invitrogen, Paisley, UK). This suspension was carefully overlayered with 1 ml DMEM and incubated at room temperature for 15 min. The upper layer was removed and spermatozoa pelleted by centrifugation (1000 × *g*) for 5 min at room temperature. Cells were washed twice by gentle centrifugation as above. For immunofluorescence studies, the re-suspended cells were smeared onto glass slides, air-dried immediately, fixed in acetone at room temperature for 1 min and stored at −20 °C until use. To prepare lysate, the swim-up spermatozoa from 4 cauda epididymi were pelleted and incubated with mixing in 100 μl of lysis buffer for 30 min on ice. Insoluble debris was removed by centrifugation (15,000 × *g*, 15 min at 4 °C) and the supernatant stored in aliquots at −80 °C.

To compare CD59b expression in unactivated and acrosome-reacted spermatozoa, the acrosome reaction was induced essentially as described (Mizuno et al., 2004). Briefly, swim-up spermatozoa (10^6^ cells/ml of DMEM) were incubated for 1 h at 37 °C with the calcium ionophore A23187 (Sigma–Aldrich) at 1 μM to induce the acrosome reaction. Control cells were incubated without ionophore. Acrosome-reacted and control spermatozoa were smeared on glass slides and immediately air-dried. To observe CD59b distribution, the smears were incubated with FITC-labeled CD59b.2. Nuclei were counterstained with DAPI (4′-6-diamino-2-phenylindole-2 HCl; 100 ng/ml final concentration; Sigma–Aldrich). On each slide, at least 100 cells were counted and the assay was carried out in triplicate.

### 2.8 Functional inhibition assay of CD59a and CD59b in mouse sperm

Spermatozoa harvested by swim-up from two epididymi, either from wild type or *cd59a*−/− mice, were washed and suspended in 2 ml DMEM. Paired aliquots (200 μl) were incubated at 37 °C with mAbs CD59a.1, CD59b.2, or isotype-matched control mAb, each at 10 μg/ml. After 4 h of incubation, the sample was immediately placed on a glass haemocytometer slide and the total number of sperm and percentage remaining motile were counted under light microscopy. This experiment was performed in triplicate.

### 2.9 Statistical analysis

All values are expressed as mean ± standard error (S.E.M.). The statistical analysis was performed by one-way ANOVA. When significant differences were observed, statistical analysis was further carried out using unpaired *t*-test between two groups. Significance between two groups was claimed when *P* < 0.05.

## 3 Results

### 3.1 CD59b mRNA is highly expressed only in testis

We have previously demonstrated that CD59a is the primary regulator of MAC assembly in mouse (Baalasubramanian et al., 2004). However, in a recent work (Qin et al., 2006), abundant expression of CD59b mRNA in a number of tissues was reported. In an attempt to clarify this issue, which is of key importance for complement studies in mice, we repeated some of the experiments carried out by Qin and co-authors using the primer pairs designed by them. Under routine conditions (25 cycles of amplification), CD59a mRNA was detected in all tissues tested while CD59b mRNA was found only in testis (Fig. 1A). Increasing the number of amplification cycles to 35 (Fig. 1B) revealed weak expression of mRNA for CD59b in liver, blood cells, heart and lung. Amplified sequence was confirmed to be CD59b by sequencing.

We next re-visited the primers used in our previous quantitative PCR analysis to assess expression of the two CD59 isoforms in different mouse tissues (Baalasubramanian et al., 2004). We had designed a primer pair that annealed to both isoforms and Taqman probes specific for either CD59a or CD59b to enable accurate quantitation. Qin et al. (2006) criticised these experiments on the basis that, while both primers used in our assay matched perfectly CD59a, each had a single internal nucleotide mismatch compared to the CD59b sequence (Table 1). They suggested, without evidence, that this mismatch favoured amplification of CD59a and caused our inability to detect CD59b in tissues other than testis and bone marrow. There is a large primer design literature that shows clearly that internal mismatches, unlike those at the 3′ end, do not significantly influence amplification (Sommer and Tautz, 1989; Kwok et al., 1990; Christopherson et al., 1997; Löffert et al., 1998). Nevertheless, we addressed further this issue by repeating our previous QPCR investigation but including a second primer pair from the same sequence matching perfectly CD59b mRNA but with a single mismatch to CD59a mRNA in the same position as in the original primer set (Table 1). Using the original primer pair that matched perfectly CD59a we obtained very similar results to those we previously published (Baalasubramanian et al., 2004). When we used the pair matching CD59b, there was a small increase in threshold cycle (Ct) for both CD59a and CD59b, likely a result of altered primer annealing temperature, but there was no difference in the calculated relative amounts for CD59a and CD59b mRNA in testis compared to the original primer set (Table 2). Of note, QPCR with either primer set did not detect any CD59b mRNA in liver, suggesting that the high cycle number PCR described above was detecting very small amounts of mRNA in these tissues. In summary, the data shows an 8-fold greater expression of CD59a mRNA in liver compared to testis, a 5-fold greater expression of CD59a mRNA compared to CD59b in testis and undetectable expression of CD59b in liver, regardless of primer set used.

In light of these results we developed a semi-quantitative PCR to quantify the low levels of CD59b mRNA detected in tissues. In order to be able directly to compare the expression of both isoforms, we designed a new primer pair within exon 4 (Table 1), which is 100% homologous to both mRNAs. Amplification of DNA-free mRNA with these primers will result in bands of 199 bp for CD59a and 162 bp for CD59b. In testis we detected both isoforms as expected (Fig. 2A). Densitometric comparison of band intensities at higher dilutions of template, when the amplification reaction is in the linear range, showed approximately 5-fold higher expression of CD59a mRNA as compared to CD59b mRNA in testis, a result compatible with the QPCR data (Table 2) and our published results (Baalasubramanian et al., 2004). However, in liver we failed to detect presence of CD59b even after 40 cycles of PCR (Fig. 2B). We reasoned that the large excess of CD59a mRNA in liver out-competes trace amounts of CD59b mRNA for limited reagents in the initial cycles of amplification, thereby reducing the chance for amplification of the low abundance CD59b mRNA. To test this reasoning we performed semi-quantitative PCR in separate tubes, using the primers specific for either CD59a or CD59b mRNA (Qin et al., 2006). Firstly, to optimise the annealing and amplification efficiency for both primer pairs, we performed this reaction for testis mRNA (Fig. 3A). Similar band intensities for CD59a and CD59b were obtained for 5 × 10^5^-fold and 10^5^-fold template dilution respectively (Fig. 3A and B). This indicated an approximate 5-fold higher expression of CD59a mRNA compared to CD59b mRNA, supporting our results described above (Table 2) and published (Baalasubramanian et al., 2004), and confirming similar amplification efficiency for the specific primer pairs. Amplification of liver mRNA using these primers, and comparison of band intensities in dilutions of templates showed that expression of CD59b mRNA in liver was approximately 10^5^-fold less compared to that of CD59a mRNA (Fig. 3C and D similar band intensities for CD59a and CD59b at 5 × 10^5^ and 5-fold dilution respectively). In these latter experiments we used liver perfused with saline at the time of sacrifice to remove the bulk of entrapped blood; nevertheless, the trace mRNA detected might be from residual blood cells, which clearly express CD59b protein at low level (Baalasubramanian et al., 2004; Qin et al., 2006). To clarify this issue, we compared mRNA from perfused and non-perfused liver by QPCR using CD59b-specific primers and found the amount of CD59b mRNA in liver was reduced 12-fold by perfusion (Fig. 3E). For comparison, expression of CD59b in testis was 2200-fold higher than in unperfused liver and approximately 25,000-fold higher than in perfused liver. Taken together these results strongly suggest that the detectable traces of CD59b mRNA in liver and likely other organs are a consequence of contamination with blood cells.

### 3.2 Expression of CD59b protein is testis restricted

We have previously reported, using immuofluorescence staining, that CD59b protein was highly expressed in testis but absent from all other organs tested (including liver, lungs, spleen, kidney and heart) (Baalasubramanian et al., 2004). We here extend these studies by Western blotting of testis, liver, lungs, plus aorta, chosen because of the suggested role of CD59 in vascular disease (Qin et al., 2004) (Fig. 4). Each organ was perfused with saline prior to preparation of protein lysates. CD59a was strongly detected in all the tissues; however, CD59b was detected only in testis lysates. These data confirm our published contention that organ expression of CD59b protein is restricted to testis.

### 3.3 Expression of CD59b mRNA in testis coincides with puberty and plays a role in spermatozoal motility

We previously reported that CD59b expression in testis was restricted to developing and mature spermatozoa (Baalasubramanian et al., 2004). To confirm this germ cell restricted pattern we examined expression of CD59b mRNA in testis from pre-pubertal mice. CD59b mRNA was absent in testes harvested from mice at days 10 and 20 post-partum and appeared only from day 30 on, coincident with puberty (Fig. 5A). In contrast, CD59a mRNA was present in testes at all timepoints. RNA extracted from embryos at days 5, 10 and 17 were all positive for CD59a but negative for CD59b mRNA (Fig. 5A). These observations were confirmed by Western blotting (Fig. 5B). Expression of CD59b protein was highest in spermatozoa, intermediate in adult testis and absent from infant testis. CD59a was present in all the lysates, albeit at low level in spermatozoa and with a reduced apparent molecular mass compared with the testis protein, suggesting modification during sperm maturation.

We previously reported that CD59b on spermatozoa was focussed on the head region in a highly granular pattern (Baalasubramanian et al., 2004). Here we have explored the expression pattern of CD59b in more detail. In freshly isolated spermatozoa, more than 80% showed this head/granular staining pattern, a minority showing a more diffuse staining on the head region (Fig. 6). CD59b was weakly expressed on spermatozoal tails and, in about two thirds, strongly in the mid-piece. Initiation of the acrosome reaction (with A23187) caused a precipitous loss of CD59b expression on sperm heads, more than 60% of cells being negative by 30 min and 90% by 180 min post-initiation, indicating that CD59b was shed with the outer acrosomal membrane (Fig. 6). These data suggested that CD59b might play a role in acrosome function, an essential component of sperm capacitation for fertilisation. Therefore, we next investigated whether ligation of CD59b with antibody influenced spermatozoal mobility, a surrogate marker for fertilisation capacity (Fig. 7). Ligation of CD59b caused a significant suppression of motility of spermatozoa harvested from both wild type and *cd59a*−/− mice. As a control, CD59a was similarly ligated but did not alter spermatozoal motility compared with the effect of a control antibody. The data suggest that CD59b but not CD59a has a role in regulating spermatozoal motility. These findings are of particular relevance in that a major feature of the CD59b knockout mouse was spermatozoal dysfunction that included diminished motility and infertility (Qin et al., 2003).

## 4 Discussion

We have recently examined the distribution patterns of the two isoforms of CD59 in the mouse and concluded, based upon its broad distribution, that CD59a is the primary regulator of MAC assembly in mouse (Baalasubramanian et al., 2004). We were unable to detect the expression of CD59b, either at mRNA or protein level, in brain, lungs, heart, liver, spleen and kidney. These data have recently been questioned by Qin et al. (2006) who first used a BLAST search of the mouse EST database and found ESTs matching the CD59b sequence from several tissues and organs. These *in silico* data were supported by RT-PCR analyses using primer sets specific for CD59a and CD59b, respectively that showed abundant expression of CD59b mRNA in all tissues tested, indeed, expression in testis was lower than in other organs. The apparent absence of CD59b mRNA in the CD59a knockout mouse in these published data was unexplained.

Here we designed a number of quantitative and semi-quantitative assays to comprehensively address this controversial issue. Our data unambiguously demonstrated that expression of CD59b is essentially restricted to testis (Figs. 3 and 4). A comparative quantitative analysis of expression of CD59b mRNA in perfused and unperfused liver (Fig. 3) showed a 12-fold decrease in expression of CD59b following perfusion, strongly suggesting that the trace detection of this mRNA was a consequence of contamination with blood cells. This would explain why Qin et al. (2001) were able to detect CD59b in multiple mouse tissues using Northern analysis in which they loaded 10 μg of mRNA in each lane, a huge excess for this sensitive procedure. The contamination likely also explains the presence in multiple tissues of CD59b-specific EST sequences.

We further demonstrated that the testis expression of CD59b coincides with puberty, supporting our findings of expression only on spermatozoa and their immediate precursors (Fig. 5). We found that CD59b was released from spermatozoa heads upon acrosome activation (Fig. 6), an observation that strongly support a role for this protein in functioning of acrosome. Ligation experiments with antibodies showed that CD59b but not CD59a was involved in spermatozoa motility (Fig. 7), providing support for an earlier report describing decreased motility and viability of sperm in *cd59b* KO mice (Qin et al., 2005).

## 5 Concluding remarks

The data presented here, obtained using a broad panel of reagents and methods designed to give unbiased and unequivocal results, show that CD59b expression is limited. CD59b mRNA is abundantly expressed only on male germ cells and present in trace amounts in bone marrow and blood cells, but is absent from other organs where trace detection of mRNA is likely due to blood contamination. CD59b protein is abundant only on developing and mature spermatozoa. Erythrocytes express CD59b at low levels that we have previously quantified as less than 200 molecules per cell, irrelevant for protection from complement when CD59a is present at 2500 molecules per cell (Baalasubramanian et al., 2004). We show a unique distribution pattern of CD59b protein on spermatozoa, the precipitous loss of this protein with outer acrosomal membranes and effects of CD59b ligation on sperm motility. We conclude that CD59a is indeed the principal regulator of MAC expressed in the mouse and that the CD59a knockout is an appropriate model for studying the roles of MAC and its regulation in disease models. The CD59b knockout mouse might prove of value for studies of fertility; however, it should be noted that the mouse described by Halperin and co-workers is, for unexplained reasons, also markedly deficient in CD59a (Qin et al., 2006), limiting its utility for studying specific roles of CD59b in vivo.

## Figures and Tables

**Fig. 1:** RT-PCR detection of CD59a and CD59b in mouse tissues. Primer pairs described in the text and specific for each isoform were used for the PCR step and either 25 (A) or 35 (B) amplification cycles were carried out. Using these primers, an approximately 350 bp product was obtained from CD59a mRNA and was readily detected in all tissues after 25 cycles. CD59b mRNA was detected after 25 cycles in testis only and the product size was approximately 400 bp. After 35 cycles of amplification, this product was detected in all tissues.

**Fig. 2:** RT-PCR analysis of expression of CD59a and CD59b using common primers. A new primer pair was designed from identical sequences within exon 4 of CD59a and CD59b mRNA and used to amplify mRNA from testis (A) and liver (B). Forty amplification cycles were carried out using different dilutions of cDNA (shown above) as template. The amplified products were 199 bp-long for CD59a and 162 bp-long for CD59b. Products were separated in 5% PAAG. Intensity of the bands was measured and the CD59a/CD59b ratio calculated from three independent experiments (given below each band pair in A). This ratio was approximately 1 when the cDNA template was not diluted or diluted 5-fold, indicating that amplification has reached saturation. However, the calculated ratio was around 5 for higher dilutions of the template, suggesting that amplification at the final point was in the linear range.

**Fig. 3:** Semi-quantitative RT-PCR to estimate relative expression of CD59a and CD59b in testis (A) and perfused liver (C). Different primer pairs for each isoform and different dilutions of the cDNA-templates (numbers above) were used. Thirty-five cycles were carried out and reaction products were separated in a 1% agarose gel. The average densitometric intensity for each band calculated from three independent experiments is given. Panels B and D present band intensity for CD59a (♦) and CD59b (■) as function of template dilution for testis and liver, respectively. (E) SYBR Green QPCR analysis of expression of CD59b in liver without and with perfusion using primers specific for CD59b. Number of the CD59b mRNA copies in liver (set as 1 for unperfused) was compared that in testis. Data are mean of two independent experiments ± S.E.M.

**Fig. 4:** Western blot for expression of CD59a and CD59b in different mouse tissues. Lysates from testis, liver, lungs, and aorta were separated by SDS-PAGE, blotted to nitrocellulose membranes, and probed either with the mAb CD59a.1 or with CD59b.2 for detection of CD59a and CD59b, respectively.

**Fig. 5:** Expression profile of CD59a and CD59b during development and testis maturation. Whole embryos were used to purify total RNA and assess expression of CD59a and CD59b. (A) A primer pair that recognizes both isoforms yielding products of 204 bp for CD59a and 237 bp for CD59b was used. EL4 cells transfected with plasmids expressing either CD59a or CD59b were used as controls. (B) Western blots analysis of CD59a and CD59b expression in infant and adult testis and sperm. Equal amounts of proteins were loaded in each lane in both panels.

**Fig. 6:** Distribution of CD59b in spermatozoa and effects of acrosome activation. The right-hand panel shows representative images for each pattern of CD59b staining with CD59b.2 mAb. Arrowheads point to the sperm head showing granular and diffuse staining respectively. Arrows indicate the mid-piece showing dense staining. The left panel shows the effects of acrosome reaction on CD59b expression. Data are means of two independent experiments ± S.E.M. Compared sets are shown by columns with interrelated *P* values for comparison (*P < 0.0001).

**Fig. 7:** Ligation of CD59a and CD59b in mouse sperm with monoclonal antibodies. In wild type (WT) and *cd59a*−/− mouse sperm, CD59a and/or CD59b were ligated with CD59a.1 or CD59b.2. Rat and mouse IgG1 were used as controls for CD59a and CD59b specific antibodies as appropriate. The percentage of sperm retaining motility at 4 h post-antibody ligation was assessed. Data shown are means of three independent experiments ± S.E.M. Compared sets are shown by columns with interrelated *P* values for comparison (*P < 0.05).

**Table 1:** Primers used for detection of Cd59a and Cd59b mRNA

Sequence detected	Primer pairs
Cd59a + Cd59b by QPCR (sequence matches Cd59a) (Baalasubramanian et al., 2004)	5′-GCCGGAATGCAAGTGTATCA-3′ (F); 5′-GTCCCCAGCAATGGTGTCTT-3′ (R)
Cd59a + Cd59b by QPCR (sequence matches Cd59b)	5′-GCCGGAAGGCAAGTGTATCA-3′ (F); 5′-GTCCCCAGCAATGCTGTCTT-3′ (R)
Cd59a (Qin et al., 2006)	5′-TGTCTAGAGCAGGATCTAGC-3′ (F); 5′-ATCCGTCACTTTTGTTACAC-3′ (R)
Cd59b (Qin et al., 2006)	5′-AGTCACTGGCGATCTGAAAAG-3′ (F); 5′-ATGAGGAAGTTTCTGCGTTG-3′ (R)
Cd59a + Cd59b (exon 4)	5′-GTTCTGGTGGCCATTTTGAA-3′ (F); 5′-TGTCCAAGATGTTCAAGTGAAC-3′ (R)
Cd59a + Cd59b (expression during testis development)	5′-GATTCCTGTCTCTATGCTGTA-3′ (F); 5′-CAAAATGGCCACCAGAAC-3′ (R)
β-Actin	5′-ACGGCCAGGTCATCACTATTG-3′ (F); 5′-AGTTTCATGGATGCCACAGGAT-3′ (R)

**Table 2:** Comparison of data from QPCR analyses obtained by primers matching either Cd59a or Cd59b

	Primers matching CD59a, Ct		Primers matching CD59b, Ct		ΔΔCt = ΔCt(b) − ΔCt(a)		Relative amount of CD59a (%)^a^		Relative amount of CD59b (%)^a^	
	CD59a	CD59b	CD59a	CD59b	Primers matching CD59a	Primers matching CD59b	Primers matching CD59a	Primers matching CD59b	Primers matching CD59a	Primers matching CD59b
Testis	24.8 ± 0.3	27.1 ± 0.4	26.1 ± 0.4	28.4 ± 0.4	2.3 ± 0.3	2.3 ± 0.4	100 ± 4	100 ± 5	20 ± 1	20 ± 1
Liver	21.8 ± 0.3	UD	23.1 ± 0.3	UD	UD	UD	822 ± 9	811 ± 8	UD	UD

UD: undetectable, Ct: threshold cycle, ΔCt(a), ΔCt(b): Ct measured for CD59a or CD59b respectively, standardised by Ct for the housekeeping gene (β-actin).

a Data are presented as percent compared to testis.
